The article "Metacognitive function in young adults is impacted by physical activity, diet, and sleep patterns" was published in 2025. Journal: PLoS One.

# Metacognitive function in young adults is impacted by physical activity, diet, and sleep patterns

**DOI:** 10.1371/journal.pone.0317253

**Published:** 2025-01-09

**Authors:** G. Kyle Gooderham, Todd C. Handy

**Affiliations:** Psychology, University of British Columbia, Vancouver, British Columbia, Canada; The University of Auckland, NEW ZEALAND

## Abstract

Our cognitive capacities like working memory and attention are known to systematically vary over time with our physical activity levels, dietary choices, and sleep patterns. However, whether our metacognitive capacities––such as our strategic use and optimization of cognitive resources––show a similar relationship with these key lifestyle factors remains unknown. Here we addressed this question in healthy young adults by examining if physical activity, diet, and sleep patterns were predictive of self-reported metacognitive status. Participants completed a set of validated surveys assessing these lifestyle factors over the past week to month, as well as three measures of metacognition. Using multiple regression and exploratory factor analyses we identified four clusters of metacognitive processes that are sensitive to lifestyle behaviours. Specifically, knowledge of and offline regulation of cognition is linked with physical activity, on-line cognitive regulation is related to diet, and metacognitive worry is associated with sleep behaviours. These findings suggest that lifestyle behaviours do not just affect objective cognitive functioning, but also the meta-level processes we use to monitor our cognitive performance and exert strategic control over our cognitive resources.

## Introduction

Our cognitive capacities are not fixed in time, but rather, have been shown to systematically vary with at least three key lifestyle behaviours (LSBs)––physical activity (PA) levels, dietary behaviours, and sleep patterns [1–3]. While the relationship between cognition and LSBs have been most intensively studied in older adults and adolescents [4–9], emerging evidence suggests that these associations also may extend to cognitively healthy young adults [10]. Cognitively healthy young adults are characterized as experiencing a period of maximal cognitive function, performance stability, and structural integrity [11] which comparative neuroimaging and behavioural measurement indicates extends from approximately 15 to 35 years of age [12–14]. For the purposes of our studies, we define young adults as those from the ages of 17 to 35.

In particular, young adults who partake in regular PA [15], who make more nutritious dietary choices [16], and get recommend levels of sleep [17] show enhanced cognitive functioning, relative to age-matched peers with less-optimal lifestyle patterns. Building on this, here we examined whether the associations between these LSBs and cognition in healthy young adults extend to *metacognitive* function, or the cognitive processes we use to monitor and adaptively control our cognitive performance [18, 19].

The question is critical because metacognitive measures capture a facet of cognition that is functionally distinct from cognitive processes per se, or what is assessed when––for example––executive, attentional, or working memory function are tested via a Stroop, Eriksen Flanker, or N-back tasks, respectively [20]. Metacognition is a fundamental cognitive ability that enables individuals to evaluate their performance on cognitive tasks and direct corrective control to engage the necessary cognitive processes [21]. Metacognition is generally accepted as comprising of monitoring and control processes that are determined by a series of subjective appraisals of one’s knowledge and ability [22]. For example, in discussing meta-reasoning, Ackerman and Thompson [23] distinguish between object-level and meta-level processing. In our study, we are concerned with how meta-level processing is affected by lifestyle behaviours. Specifically, as reviewed by Efklides [24], models of metacognition concern both the strategic use or deployment of specific cognitive processes (i.e., when an individual chooses to use a given process) and their optimization when used/deployed (i.e., how efficiently is an individual engaging or using the chosen process). As such, it remains an open question whether LSBs such as PA, diet, and sleep may be related to these vital meta-level aspects of cognition that transcend what process-specific cognitive measures are designed to assess.

Metacognitive functions influence lifestyle behaviours. For instance, recreational endurance runners reported less engagement in metacognitive processes during PA than did elite athletes, who practiced metacognitive planning, monitoring, reviewing, and evaluating of performance [25, 26]. The role of metacognition in lifestyle behaviours extends to diet and sleep behaviours as well. Dietary choices are influenced by metacognition [27] and metacognitive worry is higher in individuals with eating disorders compared to non-clinical controls [28, 29]. Furthermore, because metacognitions about sleep contribute to maladaptive sleep behaviours [30], these metacognitions can be modified to facilitate improved sleep [31]. Ultimately, metacognition is associated with lifestyle behaviours, at least insofar as metacognition contributes to the behaviours.

Less well documented is how lifestyle behaviours affect metacognition. A meta-analysis of the effects of PA on cognitive functions in children conducted by Álvarez-Bueno et al. [32] revealed that PA had a small positive effect on “higher-level executive functions” and “cognitive lifeskills,” which were combined into a general measure of metacognition. Relatedly, increased physical fitness is correlated with improved metacognitive performance, at least in obese preadolescents [33]. However, unequivocal support for lifestyle behaviours benefitting metacognitive functioning is not forthcoming. In adult populations, metacognitive monitoring of memory and learning is affected by PA interventions, though both enhancement and impairment of absolute and relative performance is observed [34]. A similar pattern was observed with aspects of diet [35]. In contrast, sleep deprivation does not affect metacognitive monitoring [36, 37], though the inability to manage performance decrement suggests failure of metacognitive control processes. The small extant literature, and heterogeneity of findings, underscores the need to address whether lifestyle behaviours are associated with metacognition.

Young adults are a demographic who may show sensitivity to lifestyle behaviours in metacognitive functioning for at least three reasons. First, young adult’s object-level cognitive functioning is responsive to changes in PA, diet, and sleep behaviours [15–17]. Second, young adults’ metacognitive monitoring and control systems are sensitive to changes in task performance at an object-level and display effective strategy implementation to correct for these changes [38]. In fact, metacognition mediates the relationship between goal directed behaviour and metacognitive, cognitive, and interpersonal resource use strategies in achieving these goals [39]. Finally, young adults and other aged populations differ in the metacognitive monitoring and control of their cognitive processes [40]. In a metamemory task, young adults and older adults differed in the metacognitive monitoring and control strategies they employed, despite commensurate knowledge retention [41]. Compared to young adults, high cognitive load tasks reduce available cognitive resources that older adults can allocate to metacognitive operations, impairing performance [42].

Towards addressing the question of whether lifestyle behaviours are associated with metacognitive functioning in young adults, our study design reflected three specific goals. First, we wanted to establish the extent to which PA levels, dietary habits, and sleep patterns are each associated with metacognitive function in healthy young adults. Second, with an initial baseline established, we wanted to determine whether the data pattern could be replicated in a second sample. Finally, given the interdependence of PA, diet, and sleep [43–45], we wanted to control for and identify the individual effects of each.

## Study One

Study One was conducted to assess the relationship between PA, diet, and sleep with three measures of metacognition.

## Materials and methods

A total of 1702 participants were recruited from the University of British Columbia Department of Psychology’s Human Subject Pool. The samples were drawn from students enrolled in the Human Subject Pool’s Spring 2021 data collection period. Participants provided written informed consent prior to the beginning of data collection and were remunerated with course credit regardless of their consent status. The University of British Columbia Behavioural Research Ethics Board provided ethical approval for the study program, certificate H19-02890.

**Methods.** Participation in the study was entirely online and did not require interaction with the research team. Once recruited and enrolled in the study through the Human Subject Pool system, participants were provided with a link to the survey, hosted on the online survey tool Qualtrics. The survey, which was completed on the participants personal device(s), led respondents through three principal stages. First, having read a brief description of the study and its purpose, participants were asked to provide informed consent. Next, a series of demographic questions were completed. Finally, participants were presented with survey blocks of each of the predictor and response variables, presented in random, intermixed order.

Data analysis was conducted in R and included measure scoring, cleaning, and outlier identification and rejection. The scoring of each measure followed the protocol provided in the manuscripts describing the measure. Response outliers on the predictor variables were detected using Tukey’s fences method. This procedure identifies observations exceeding 1.5 times the interquartile range below Q1 or above Q3 as outlying data points, which are subsequently removed. Additionally, longstring analysis was performed to identify and remove respondent data if the same response option was provided consecutively for more than 90% of the length of the measure. For example, the Inventory of Metacognitive Self-Regulation (IMSR) consists of 32 questions, therefore if a respondent provided the same response for more than 28.8 consecutive questions they were removed from further analysis. Further, observations were removed based on missingness of variable scores from individual analyses.

### Materials

The measures utilized in this study have been categorized here as either predictor or response variables, depending on their purpose in data analysis. Regression models included participant’s age, sex, perceived stress, dietary habits, sleep quality, and PA as predictor variables. Subscales of the IMSR, Meta-Cognitions Questionnaire (MCQ), and Metacognitive Awareness Inventory (MAI) served as the response variable in each model.

*Participant demographics*. Respondents completed a demographic battery indicating, amongst other items, their age and sex.

*International Physical Activity Questionnaire*. The International Physical Activity Questionnaire is a self-reported measure of PA. Respondents are prompted to report their PA during the past seven days across occupational, transportation, domestic, and leisure domains. The scoring protocol provides for the calculation of Metabolic Equivalent of Task (MET) values corresponding to the exertion required to complete the task, with larger MET values indicating more PA across the assessed domains [46]. The International Physical Activity Questionnaire has high validity and reliability [47, 48], with satisfactory psychometric properties in young adult populations [49].

*Perceived Stress Scale 10*. The Perceived Stress Scale 10 is a revised version of Cohen et al’s. [50] self-report measure of appraised stress [51]. Respondents are asked to indicate the frequency with which they felt or thought a certain way in response to ten life stressors, with high scores indicating greater degrees of perceived stress. The Perceived Stress Scale 10 is a widely used measure of stress and, despite concerns over the number and organization of factors [52], is found to have satisfactory reliability and convergent validity with more comprehensive measures of stress in young adults [53].

*Pittsburgh Sleep Quality Index*. The Pittsburgh Sleep Quality Index is a self-reported measure of sleep quality in the preceding month [54]. Participants are asked to provide information pertaining to sleep efficiency, trouble sleeping, and interference on other tasks because of poor sleep. From these questions a composite score is computed, with higher scores indicating worse sleep quality. The Pittsburgh Sleep Quality Index has demonstrated good reliability and validity in a meta-analysis of thirty-seven studies of clinical and non-clinical samples [55].

*Rapid Eating and Activity Assessment for Participants Short Version*. The Rapid Eating and Activity Assessment for Participants Short Version is a sixteen-item self-report measure of an individual’s dietary habits [56]. Respondents are prompted to indicate the frequency of achieving certain dietary thresholds, such as meeting daily consumption of servings of fruit and vegetables, in an average week. Thirteen of the items are scored on a likert scale with response options of Does not apply to me, Rarely/Never, Sometimes, and Usually/Often, corresponding to scores of 3, 3, 2, and 1. The scores on these items are summed, with higher scores indicating healthier dietary habits. The Rapid Eating and Activity Assessment for Participants Short Version has shown good validity when compared with more comprehensive measures of dietary habits in young adults [56] in addition to a positive correlation with chemical indices of diet quality [57].

*Inventory of Metacognitive Self-Regulation*. The IMSR is a thirty-two-item self-reported measure of “metacognitive awareness and regulatory skills in a problem-solving context” [58]. Comprising of knowledge of cognition, objectivity, problem representation, subtask monitoring, and evaluation subscales, this questionnaire probes participants on the frequency in which they engage in problem solving activities. *I try to understand what the problem is asking me*, from the Problem Understanding subscale, captures the intention of the measure. The IMSR has satisfactory psychometric properties [58].

*Meta-Cognitions Questionnaire*. The MCQ is a sixty-five item self-reported measure of beliefs about worry and intrusive thoughts [59]. The MCQ assesses five aspects of metacognition: positive beliefs about worry; negative beliefs about the uncontrollability of thoughts and corresponding danger; lack of cognitive confidence; negative beliefs about thoughts in general, including themes of superstition, punishment, and responsibility; and cognitive self-consciousness. Respondents indicated their agreement with items on a four-point likert scale, with higher values indicating greater endorsement. The MCQ demonstrates satisfactory reliability and validity in young and middle aged adult samples [59].

*Metacognitive Awareness Inventory*. The MAI is a fifty-two-item self-reported measure of an individual’s knowledge and regulation of cognition in a learning context [60]. The knowledge of cognition subscale comprises aspects of declarative, procedural, and conditional knowledge, while the regulation of cognition subscale consists of planning, information management, monitoring, debugging, and evaluation processes. Participants are prompted to indicate how typical it is for them to employ different learning strategies and behaviours on a five-point likert scale, with higher scores signalling more common use. Psychometric evaluation of the MAI demonstrates the inventory as having good reliability and validity in young adult populations [60].

### Results

The purpose of these investigations was to determine the effects of LSBs on metacognitive functioning, while accounting for basic demographic information. To accomplish this, we utilized a consistent methodological approach with LSBs and demographic factors serving as predictor variables and a measure of metacognition as the response variable in multiple regression analyses.

Participants completed each of the predictor variables and one of the metacognitive response variables. Respondents were retained in the dataset if they consented to the study, provided demographic information included in the analyses, and were not identified as outliers. As a result, 43 of the 536 participants who completed the IMSR, 54 of the 577 participants who completed the MCQ, and 60 of the 589 participants who completed the MAI were removed from further analysis, leaving final samples of 493, 523, and 529 respectively.

Descriptive statistics of the participant demographics and predictor variables for each dataset, as well as an indicator of the internal consistency of the response variables (Cronbach’s alphas), are available in Table 1. See Table 2 for beta-weights and model fit. Variance inflation factors were calculated for each model due to the potential for collinearity between predictors within the regression models. All variance inflation factors were within the acceptable range (<1.5).

**Table 1:** Descriptive statistics for Studies One and Two.

			Study One												Study Two			
			*n*	*M*	*SD*	*α*	*n*	*M*	*SD*	*α*	*n*	*M*	*SD*	*α*	*n*	*M*	*SD*	*α*
Predictor Variables																		
	Age		493	20.79	2.01		523	20.93	2.21		529	20.99	2.20		564	20.87	2.47	
	Sex		493				523				529				564			
		Female	382				412				413				438			
		Male	111				111				116				126			
	IPAQ		461	3001.89	2663.65		488	2907.41	2726.88		479	2834.97	2654.77		524	3805.22	3383.28	
	PSS		455	20.99	6.29		487	20.51	6.40		507	20.28	6.26		535	21.35	5.89	
	PSQI		462	7.16	3.22		495	6.79	3.17		504	6.94	3.18		533	7.34	3.20	
	REAP-S		430	30.37	4.30		480	30.58	4.17		506	30.68	4.37		531	29.60	4.47	
Response Variables																		
	Inventory of Metacognitive Self-Regulation																	
		Evaluation	451	22.53	4.53	.89									482	22.41	4.33	.88
		Subtask Monitoring	451	21.80	3.56	.80									479	21.70	3.88	.83
		Objectivity	455	19.26	4.21	.80									486	19.12	4.08	.80
		Problem Representation	457	19.93	3.15	.79									483	19.56	3.30	.83
		Knowledge of Cognition	451	20.79	3.59	.74									476	20.77	3.64	.75
	Meta-Cognitions Questionnaire																	
		Positive Beliefs					457	35.47	10.14	.92					461	38.09	10.53	.92
		Uncontrollability and Danger				467	36.96	11.33	.94					466	39.10	10.90	.93
		Cognitive Confidence					467	19.12	6.12	.88					470	20.39	6.17	.87
		Negative Beliefs					473	26.06	7.05	.86					465	26.76	7.33	.87
		Cognitive Self-Consciousness				476	18.66	4.04	.78					476	19.24	4.11	.81
	Metacognitive Awareness Inventory																	
		Knowledge of Cognition									486	59.63	10.11	.91	511	59.21	10.10	.91
		Declarative Knowledge									488	28.61	4.82	.83	513	28.24	4.96	.82
		Procedural Knowledge									490	13.82	2.84	.76	517	13.79	2.79	.76
		Conditional Knowledge									489	17.15	3.40	.74	515	17.17	3.26	.75
		Regulation of Cognition									485	112.50	19.53	.94	513	112.06	18.47	.94
		Planning									491	22.21	4.86	.81	515	22.20	4.54	.77
		Information Management									487	31.15	5.72	.82	517	30.89	5.28	.80
		Monitoring									504	22.43	4.97	.82	532	22.33	4.80	.81
		Debugging									505	18.37	3.37	.75	532	18.21	3.22	.71
		Evaluation									489	18.53	4.23	.77	516	18.28	4.09	.74

*Note*. Study One consisted of three different samples. IPAQ = International Physical Activity Questionnaire; PSS = Perceived Stress Scale 10; PSQI = Pittsburgh Sleep Quality Index; REAP-S = Rapid Eating and Activity Assessment for Participants Short Version.

**Table 2:** Regression results for Study One.

* *		IMSR									MCQ										MAI																			
		Evaluation	Subtask Monitoring		Objectivity		Problem Representation		Knowledge of Cognition		Positive Beliefs		Uncontrollability and Danger		Cognitive Confidence		Negative Beliefs		Cognitive Self-consciousness		Declarative Knowledge		Procedural Knowledge		Conditional Knowledge		Planning		Information Management Strategies		Monitoring		Debugging Strategies		Evaluation		Knowledge of Cognition		Regulation of Cognition	
Intercept	*β*	.04	.03		-.06		.10		.02		-.06		-.02		-.07		-.09		-.07		.02		.04		.02		.03		.01		-.03		.05		-.03		.02		.01	
Age	*β*	.07	.07		.07		.10		.02		-.06		-.03		-.15	**	-.15	**	-.13	*	.02		.01		-.01		.05		.06		.10	*	-.03		.09		.01		.08	
Sex	*β*	-.23	-.13		.11		-.28	*	-.10		.11		.01		.13		.27	*	.21		-.14		-.15		-.17		-.21		-.09		-.01		-.27	*	.07		-.17		-.11	
IPAQ	*β*	.05	.08		.11	*	.10		.10	*	.05		.02		-.01		.06		.06		.12	*	.10	*	.20	***	.15	**	.17	***	.17	***	.13	**	.17	***	.15	**	.18	***
PSS	*β*	-.03	-.15	*	-.05		-.05		-.30	***	.15	**	.54	***	.35	***	.33	***	.12	*	-.33	***	-.35	***	-.32	***	-.36	***	-.22	***	-.19	***	-.19	***	-.14	*	-.36	***	-.26	***
PSQI	*β*	-.07	.01		-.05		.10		-.01		.04		.10	*	.08		.08		.12	*	.04		.04		.05		.01		-.01		.06		.04		-.04		.05		-.01	
REAP-S	*β*	-.07	-.03		-.01		-.03		.06		-.02		-.06		-.10	*	-.04		-.01		.00		.00		.00		.03		.03		.07		.05		.00		.00		.03	
Model Fit	*RSE*	0.99	0.99		1.01		0.95		0.92		0.99		0.80		0.88		0.90		1.00		0.96		0.96		0.97		0.95		0.98		0.98		0.98		0.99		0.95		0.97	
	*R* ^2^	.02	.03		.03		.04		.11		.04		.38		.21		.18		.06		.11		.11		.12		.14		.08		.07		.06		.06		.13		.10	
	*F*	1.30	1.96		1.87		2.21		7.71		2.44		40.06		17.59		14.10		4.09		8.39		9.07		9.98		11.72		6.38		5.58		4.59		4.53		10.64		8.19	
	*p*	.256	.070		.086		.042		.000		.025		.000		.000		.000		.001		.000		.000		.000		.000		.000		.000		.000		.000		.000		.000	
	*N*	374	372		374		376		372		392		398		400		403		406		432		434		434		435		433		444		445		434		431		431	

Note.

* p < .05.

** p < .01.

*** p < .001. IPAQ = International Physical Activity Questionnaire; PSS = Perceived Stress Scale 10; PSQI = Pittsburgh Sleep Quality Index; REAP-S = Rapid Eating and Activity Assessment for Participants Short Version; IMSR = Iventory of Metacognitive Self-Regulation; MCQ = Meta-Cognitions Questionnaire; MAI = Metacognitive Awareness Inventory.

#### Inventory of Metacognitive Self-Regulation

PA was predictive of Objectivity, *β* = 0.11, 95% CI [0.007, 0.22], *t*(367) = 2.09, *p* = .04, and Knowledge of Cognition, *β* = 0.10, 95% CI [0.00, 0.20], *t*(365) = 1.97, *p* = .05, such that more physically active young adults reported higher objectivity and knowledge of cognition. In addition, PA was marginally predictive of the Problem Representation subscale, *β* = 0.10, 95% CI [-0.003, 0.20], *t*(369) = 1.92, *p* = .06.

In addition, perceived stress significantly predicted the Subtask Monitoring and Knowledge of Cognition subscales, with more perceived stress linked to worse metacognitive performance. Neither sleep nor diet were significantly predictive of any subscales of the IMSR.

Finally, the model explained a significant proportion of variance on the Problem Representation and Knowledge of Cognition subscales.

#### Meta-Cognitions Questionnaire

PA was not associated with any of the subscales of the MCQ.

Rather, diet was linked to the Cognitive Confidence subscale, *β* = -0.10, 95% CI [-0.20, -0.01], *t*(393) = -2.17, *p* = .03, while sleep was predictive of Uncontrollability and Danger, *β* = 0.10, 95% CI [0.007, 0.19], *t*(391) = 2.12, *p* = .04, and Cognitive Self-Consciousness, *β* = 0.12, 95% CI [0.008, 0.24], *t*(399) = 2.11, *p* = .04, subscales. Furthermore, perceived stress was significantly predictive of each subscale of the MCQ. In all instances, worse diet, sleep, or perceived stress scores were associated with negative metacognitive outcomes.

The model explained a significant proportion of variance for each of the MCQ’s subscales.

#### Metacognitive Awareness Inventory

Both PA and perceived stress were significantly predictive of every component of metacognition as assessed by the MAI. Participants with higher PA levels or lower stress reported greater metacognitive functioning.

Neither dietary nor sleep habits were linked to any of the subscales of the MAI.

The model explained a significant proportion of variance for each subscale of the MAI.

### Discussion

We observed significant relationships between our variables of interest and dimensions of metacognition. Young adults who engaged in higher levels of PA reported better metacognitive processing. Further, while the combination of LSBs explained metacognitive performance, we also note a general trend where only one LSB was significantly related to the measure of metacognition. Therefore, though the effects of LSBs may be additive in affecting metacognition, specific behaviours have specific benefits.

Nevertheless, two questions limit the interpretability of Study One. First, given the findings, can they be replicated? Second, are the differential associations between LSBs on the three measures of metacognition because these factors are affected differently or due to between-subject variance that the study did not control for? We conducted Study Two as a within-subjects design to address these concerns.

## Study Two

Study Two followed sequentially from Study One and employed the same materials and methods.

## Materials and methods

Participants were recruited from the University of British Columbia Department of Psychology’s Human Subject Pool during the Spring 2022 data collection period. Of the initial sample of 626 participants, 62 were removed from the dataset because they did not consent to the study procedures, provided incomplete responses, or were identified as inattentive or outlying respondents, resulting in a final sample of 564. All participants were granted course credit for their enrolment in the study. The University of British Columbia Behavioural Research Ethics Board provided ethical approval for the study program, certificate H19-02890.

### Methods

Study Two was conducted in the same manner as Study One. Participants were recruited from the Human Subject Pool to complete an online survey which probed them on demographic factors, LSBs, and self-reported metacognitive function. Data analysis followed and was conducted in R using primarily the psych, lavaan, and stats packages. As with Study One, longstring analysis with a 90% threshold was used to identify and remove careless or inattentive respondents.

#### Materials

Study Two consisted of a single dataset including the predictor variables as well as all three metacognitive measures described in Study One.

### Results

Analysis followed the same procedures as Study One. See Table 1 for descriptive statistics and Table 3 for beta-weights and model fit. Variance inflation factors were calculated for each model due to the potential for collinearity between predictors within the regression models. All variance inflation factors were within the acceptable range (<1.5).

**Table 3:** Regression results for Study Two.

		IMSR									MCQ										MAI																		
		Evaluation		Subtask Monitoring	Objectivity		Problem Representation		Knowledge of Cognition		Positive Beliefs		Uncontrollability and Danger		Cognitive Confidence		Negative Beliefs		Cognitive Self-consciousness		Declarative Knowledge		Procedural Knowledge		Conditional Knowledge		Planning		Information Management Strategies		Monitoring		Debugging Strategies		Evaluation	Knowledge of Cognition		Regulation of Cognition	
Intercept	*β*	.03		.03	-.04		.04		-.01		-.05		-.01		-.03		-.10		-.03		.02		.00		-.02		-.03		.01		-.03		.00		-.03	.01		-.03	
Age	*β*	-.08		-.05	-.06		-.06		-.04		-.20	***	-.04		-.11	*	-.16	***	.03		-.07		-.06		-.09		-.03		-.01		-.06		-.09		-.08	-.08		-.05	
Sex	*β*	-.05		-.16	.16		-.10		-.06		.10		-.08		.11		.31	**	.09		-.17		-.11		-.11		.00		-.15		.04		-.07		.05	-.16		-.02	
IPAQ	*β*	-.01		.05	.10	*	-.02		.10	*	.08		.03		-.03		.05		.04		.13	**	.16	***	.17	***	.12	**	.10	*	.14	**	.11	*	.05	.16	***	.13	**
PSS	*β*	.02		-.03	-.15	**	.02		-.15	**	.09		.48	***	.27	***	.34	***	.17	**	-.19	***	-.11	*	-.15	**	-.14	**	-.08		-.07		-.02		-.09	-.17	***	-.10	*
PSQI	*β*	-.06		.03	.02		.02		.09		.07		.11	*	.12	*	.03		.09		.00		-.04		.00		-.09		-.08		.00		-.01		-.05	-.01		-.07	
REAP-S	*β*	.15	**	.09	.05		.12	*	.10		-.05		-.01		-.04		-.09		.05		.10		.03		.11	*	.05		.00		.14	**	.14	**	.03	.10	*	.06	
Model Fit	*RSE*	0.98		1.00	0.98		1.00		0.98		0.96		0.83		0.93		0.90		0.99		0.96		0.97		0.96		0.97		0.98		0.98		0.99		0.99	0.95		0.98	
	*R* ^2^	.03		.02	.05		.02		.05		.07		.32		.15		.19		.05		.08		.05		.09		.07		.03		.06		.05		.03	.09		.05	
	*F*	2.55		1.39	3.38		1.33		3.54		4.88		32.50		11.80		16.09		3.45		6.79		4.32		7.09		5.51		2.65		4.66		3.77		1.98	7.28		3.89	
	*p*	.020		.218	.003		.243		.002		.000		.000		.000		.000		.002		.000		.000		.000		.000		.016		.000		.001		.068	.000		.001	
	*N*	436		434	440		437		430		415		423		426		420		430		464		468		466		466		468		482		482		467	462		465	

Note.

* p < .05.

** p < .01.

*** p < .001. IPAQ = International Physical Activity Questionnaire; PSS = Perceived Stress Scale 10; PSQI = Pittsburgh Sleep Quality Index; REAP-S = Rapid Eating and Activity Assessment for Participants Short Version; IMSR = Iventory of Metacognitive Self-Regulation; MCQ = Meta-Cognitions Questionnaire; MAI = Metacognitive Awareness Inventory.

#### Inventory of Metacognitive Self-Regulation

PA was significantly predictive of the Objectivity, *β* = 0.10, 95% CI [0.003, 0.19], *t*(433) = 2.02, *p* = .04, and Knowledge of Cognition subscales, *β* = 0.10, 95% CI [0.006, 0.19], *t*(423) = 2.09, *p* = .04. In both cases, participants with higher PA levels reported greater metacognitive performance.

As well, perceived stress was significantly associated with the Objectivity and Knowledge of Cognition subscales, such that more perceived stress impaired functioning. Additionally, better dietary habits were linked with higher reported functioning of the Evaluation and Problem Representation subscales. However, sleep was not related to any of the IMSR subscales.

Lastly, the model explained a significant proportion of variance for the Evaluation, Objectivity, and Knowledge of Cognition subscales.

#### Meta-Cognitions Questionnaire

PA was not significantly related to any of the MCQ’s subscales.

Perceived stress was significantly predictive of scores on all but the Positive Beliefs subscales, with more perceived stress impairing metacognitive functioning. In addition, sleep was linked with the Uncontrollability of Danger and Cognitive Control subscales, with worse sleep habits correlating with negative metacognitive outcomes. Nevertheless, diet was not associated with any of the subscales of the MCQ.

The model explained a significant proportion of variation of each of the MCQ’s subscales.

#### Metacognitive Awareness Inventory

PA was significantly predictive of every subscale of the MAI excepting for the Evaluation Subscale, such that higher PA levels were correlated with better metacognitive functioning.

Both perceived stress and diet were consistently significantly related to subscales of the MAI, where more perceived stress or worse dietary habits were associated with negative metacognitive outcomes. However, sleep was not predictive of scores on the MAI subscales.

Apart from the Evaluation subscale, the model explained a significant proportion of variance for each subscale of the MAI.

#### Exploratory factor analysis

To assist in interpretation of the findings of Study One and Two, which identified both significant and nonsignificant associations between LSBs and metacognition, we conducted an exploratory factor analysis of the metacognitive measure subscales to determine whether the observed significant relationships corresponded to the clustering of similar aspects of metacognition.

Measure subscales were selected as the primary unit of investigation in the exploratory factor analysis. A Pearson correlation matrix of the subscale scores for each of the IMSR, MCQ, and MAI was calculated. A Kaiser-Meyer-Olkin measure of sampling adequacy indicated overall suitability of the dataset for proceeding with an exploratory factor analysis, KMO = .91, [61], as did Bartlett’s test of sphericity, χ^2^ (153) = 4640.35, *p* < .001.

Visual inspection of the Eigenvalue scree plot suggested a four-factor model, which was then substantiated by Velicer’s minimal average particles test and parallel analysis.

The analysis was conducted with the psych::fa function in R. We selected a minimum residual factoring method with oblimin factor rotation to generate our model estimates. We surmised that oblique rotation was warranted insofar as each measure is assessing metacognition [62]. Thus, whether subscales were capturing the same dimension of cognition or not, these items should be at least moderately correlated.

Analysis loaded the subscales into factors pertaining to knowledge of cognition, metacognitive worry, online cognitive regulation, and offline cognitive regulation. Measures of model fit suggested modest model fit (eg. TLI = .91, RMSEA = .09; [63]). For factor loadings, as well as total and common variances, see Table 4.

**Table 4:** Factor analysis results for Study Two.

	Factor Loading			
	1	4	3	2
Evaluation	-.09	.15	**.75**	-.01
Subtask Monitoring	.27	.14	**.58**	-.03
Objectivity	-.05	**.71**	.24	-.04
Problem Representation	.02	-.08	**.86**	.01
Knowledge of Cognition	**.65**	.05	.16	-.07
Positive Beliefs	-.07	.29	-.08	**.56**
Uncontrollability and Danger	.12	-.23	.06	**.79**
Cognitive Confidence	-.14	-.03	-.08	**.59**
Negative Beliefs	-.09	.12	-.03	**.88**
Cognitive Self-consciousness	.25	-.12	.19	**.49**
Declarative Knowledge	**.92**	-.08	.03	-.08
Procedural Knowledge	**.80**	.09	.02	.06
Conditional Knowledge	**.80**	.18	-.07	.02
Planning	.34	**.53**	.08	.02
Information Management Strategies	**.57**	.21	.13	.08
Monitoring	.23	**.71**	.06	.04
Debugging Strategies	.32	.24	**.35**	.09
Evaluation	.14	**.75**	-.03	.01

Organizing the results of the regression analysis by the four-factor model highlight an interesting data pattern. PA is associated with knowledge of and offline regulation of cognition but not with task concurrent cognitive regulation or metacognitive worry. Additionally, sleep is linked with two measures of metacognitive worry. Finally, diet predicted three of the four measures of online cognitive regulation. To be clear, the intention of the present studies is not to derive or evaluate theoretical models of metacognition but rather to utilize available statistical approaches to better characterize and interpret the relationships between LSBs and metacognitive function. For factor loadings and beta-weights see Table 5.

**Table 5:** Beta weights by factors in Study Two.

			Factor Loading	*β*					
				IPAQ		PSQI		REAP-S	
Factor 1: Knowledge of Cognition									
	IMSR	Knowledge of Cognition	.65	.10	*	.09		.10	
	MAI	Declarative Knowledge	.92	.13	**	.00		.10	
	MAI	Procedural Knowledge	.80	.16	***	-.04		.03	
	MAI	Conditional Knowledge	.80	.17	***	.00		.11	*
	MAI	Information Management Strategies	.57	.10	*	-.08		.00	
Factor 2: Offline Regulation of Cognition									
	IMSR	Objectivity	.71	.10	*	.02		.05	
	MAI	Planning	.53	.12	**	-.09		.05	
	MAI	Monitoring	.71	.14	**	.00		.14	**
	MAI	Evaluation	.75	.05		-.05		.03	
Factor 3: Online Regulation of Cognition									
	IMSR	Evaluation	.75	-.01		-.06		.15	**
	IMSR	Subtask Monitoring	.58	.05		.03		.09	
	IMSR	Problem Representation	.86	-.02		.02		.12	*
	MAI	Debugging Strategies	.35	.11	*	-.01		.14	**
Factor 4: Metacognitive Worry									
	MCQ	Positive Beliefs	.56	.08		.07		-.05	
	MCQ	Uncontrollability and Danger	.79	.03		.11	*	-.01	
	MCQ	Cognitive Confidence	.59	-.03		.12	*	-.04	
	MCQ	Negative Beliefs	.88	.05		.03		-.09	
	MCQ	Cognitive Self-consciousness	.49	.04		.09		.05	

Note.

* p < .05.

** p < .01.

*** p < .001. IPAQ = International Physical Activity Questionnaire; PSQI = Pittsburgh Sleep Quality Index; REAP-S = Rapid Eating and Activity Assessment for Participants Short Version; IMSR = Iventory of Metacognitive Self-Regulation; MCQ = Meta-Cognitions Questionnaire; MAI = Metacognitive Awareness Inventory.

## Discussion

We investigated whether LSBs were predictive of self-reported metacognitive status. Participants completed a set of validated surveys assessing LSBs associated with PA, diet, and sleep over the past week to month. Using multiple regression and exploratory factor analyses we identified which LSBs were associated with metacognition as well as identified broader clusters of metacognitive functions that may be sensitive to health behaviours. We observed that individuals who described themselves as more physically active indicated better metacognitive knowledge of their cognitive capabilities. As well, the ability to regulate and monitor cognitive processes before, during, and after a complex cognitive task was reported as better in more physically active young adults. Still, physical activity was not related to ongoing regulation and monitoring of cognitive performance nor worry about cognition. With respect to diet, unlike more physically active young adults, neither knowledge of cognitive capabilities nor offline cognitive regulation were linked to healthier diets. Instead, young adults who reported healthful diets indicated enhanced ability to regulate and monitor their cognitive processes during complex tasks. Finally, individuals with poorer sleep habits expressed greater worry about their cognitive functioning and performance, but not with the knowledge of their cognitive functioning nor their regulation and monitoring of cognitive processing. These observations provide convergent evidence that LSBs are associated with metacognition and support the conclusion that more healthful behaviours in young adults are linked with better self-reported metacognitive functioning. Given this conclusion, several key issues and questions follow.

First, contrary to claims that cognition in young healthy individuals is not labile to LSBs [64], our findings suggest that they can be. This is important for two reasons. First, not only can young adults’ cognitive functioning be enhanced, despite being at the zenith of developmental health and performance [12], but LSBs are predictive of these outcomes. This demonstrates that cognitive function in otherwise healthy young adults who should be at their developmental peak are in fact not. Rather, it implies that the development trajectory can be modified, even in high performance states. Second, modulation of cognitive functioning may not be well captured by the behavioural measures that are paradigmatic of this line of research. Instead, consideration for the multifaceted nature of cognition, and how changes to cognitive status may be manifest, illuminates the complexity of the relationship between cognition and the body.

Second, why might metacognition be labile to LSBs where other indices of cognition are not? In response to this query, we distinguish between cognitive processes and the systems that strategically employ or harness these processes to meet specific cognitive demands [19]. We propose that while mechanistic function may remain rather stable in young, healthy adults despite variability in key LSBs, lifestyle variability may have a more pronounced and measurable impact on the use and deployment of those cognitive resources. If so, this predicts LSBs should also have a measurable influence on subjective measures of cognitive function. Further, in this way metacognition could serve as an important mediator for the relationship between LSBs and objective measures of cognitive functioning [65].

Third, distinctive metacognitive functions are differentially associated with LSBs. Specifically, knowledge of and offline regulation of cognition is linked with PA, metacognitive worry is associated with sleep habits, and online cognitive regulation is related to diet. That is to say that PA, diet, and sleep, when controlling for each other, uniquely contribute to the functioning of distinct metacognitive processes. This is analogous to objective indices of cognitive functioning where PA [66–68], sleep [2, 69], and dietary behaviours [70] provide function specific, rather than domain general, effects. While the reasons for this cannot be ascertained by the current study, we suggest that metacognitive functions are sensitive to the different neurological mechanisms by which LSBs interact with the brain. Further, these findings reinforce that metacognition is a collective suite of functions, independent of mechanistic cognitive processes, which can be independently targeted with health behaviour interventions.

Finally, public health messaging targeting young adults should underscore the importance of metacognition, and cognition generally, as well as how LSBs can enhance their performance. Health promotion in this population is critical for two reasons. First, health habits are established in young adulthood [71] and have significant consequences for health, both physically and psychologically, in later life [72]. Therefore, promoting health-positive behavioural patterns in young adults is critical for maintaining health in adulthood. Second, metacognition and LSBs exhibit a symbiotic relationship. While LSBs predict metacognitive functioning, metacognition predicts participation in health behaviours [73]. Together, public health messaging emphasizing the bidirectional relationship between metacognition and LSBs could provide the short- and long-term benefits required for lifelong healthy habit formation [74, 75].

Three limitations of the present studies inform future directions. First, though we show that lifestyle behaviours and metacognition are covariates, it would be inappropriate to infer a causal relationship. The direction of the relationships cannot be determined from the research design, and it is conceivable that cognitive variables are determinants of participation in lifestyle behaviours. In fact, the metacognitive strategies of deliberate practice, procedural knowledge, attention, and automaticity assist in skill acquisition and expert performance in physical activities [76–78], metacognitions about diet contribute to maladaptive dietary behaviours [79], and metacognitive worry is associated with impaired sleep patterns [80]. Experimental research designs could be implemented to determine the causal nature of the relationship between lifestyle behaviours and the cognitive variables observed here.

Second, the conclusions presented here are drawn from self-reported variables. These self-reported variables, including measures of both cognition and lifestyle behaviours, are liable to deviations from objective indices. Cognitive biases, inclusive of memory failures and response sets, along with self-report biases, contribute to apprehension about their use in research [81]. However, these concerns should not discount their employment, particularly if the assessment tools are well validated [82]. The validated self-report measures utilized here are suitable for assessing engagement in lifestyle behaviours as well as the metacognitive processes under investigation. Still, the use of more intensive self-report measures, device assisted assessments, or behavioural testing would allow for a depth of analysis that was not attainable in the present works. Given the limitations of each method of data collection, it would be prudent to combine self-report and objective measures, recognizing that neither is a perfect quantification of such complex constructs [83].

Finally, sampling procedures contributed to the determination of total sample size as well as the quantity and relationships between the lifestyle behaviour variables. With respect to sample size, two factors affected final study enrolment. First, we estimated small effect sizes and used those to perform *a priori* power analyses. We then modestly increased the targeted sample size to account for unusable data. Second, the University of British Columbia Department of Psychology offers, as remuneration for participating in the Human Subject Pool, research experience credits that students may apply towards their course grade. With the COVID-19 restrictions that were imposed during the Spring 2021 and Spring 2022 semesters, researchers were requested to provide more online opportunities to students so that they may still earn the course credits. Consequently, though we met our target sample sizes, we did not limit the number of respondents and were able to collect a robust sample drawn from the Human Subject Pool. Additionally, we observed statistically significant differences in lifestyle behaviours between our Spring 2021 and Spring 2022 samples. The data collected in Spring 2021, saw lower physical activity levels, *F*(3, 1948) = 12.45, *p* < .001, but better dietary patterns, *F*(3, 1943) = 6.56, *p* < .001, and sleep behaviours, *F*(3, 1990) = 2.92, *p* < .001, than in Spring 2022. While these differences should be mitigated by the data analysis procedures, it does indicate that, at baseline, the samples differed.
